RETRACTED

# Effects of Quadruple Therapy Combined with Probiotics on *Helicobacter Pylori*-Related Peptic Ulcer

**DOI:** 10.1155/2022/1221190

**Published:** 2022-10-11

**Authors:** Ye Zhou, Tingzan Li

**Affiliations:** Department of Gastroenterology, BenQ Medical Center, The Affiliated BenQ Hospital of Nanjing Medical University, Nanjing, China 210019

## Abstract

The present study was designed to observe the effect of quadruple therapy combined with probiotics on *Helicobacter pylori*-related peptic ulcer. The patients in the control group (*n* = 90) were given regular quadruple therapy including proton pump inhibitor ilaprazole enteric-coated tablet + two antibiotics amoxicillin dispersible tablet and metronidazole tablet + colloidal bismuth pectin capsule for 2 weeks. Patients in the study group (*n* = 90) were given abovementioned quadruple therapy combined with probiotics live combined *Bifidobacterium*, *Lactobacillus*, and *Enterococcus* Capsules, oral for 2 weeks. Then Hp clearance rate, recurrence rate, levels of gastrointestinal hormone makers, and advance reactions between two groups were compared. At the 2nd week after the treatment, the *Helicobacter pylori* clearance rate in the study group (87.79%) was significantly higher than the control group (78.89%), and the total recurrence rate in the study group (6.67%) was significantly lower than the control group (13.33%) (*P* < 0.05). Serum gastrin and motilin expression were lower, and somatostatin expressions was significantly higher than those in the control group (*P* < 0.05). There was no significant difference in the total incidence of adverse reactions between the two groups (*P* > 0.05). In summary, quadruple therapy combined with probiotics in the treatment of *Helicobacter pylori*-related peptic ulcer can improve the *Helicobacter pylori* clearance rate, reduce the *Helicobacter pylori* recurrence rate, and is beneficial to improving the level of gastrointestinal hormones, with certain safety.

## 1. Introduction

The peptic ulcer has the characteristics of a long course, difficulty of curing, easy recurrence, etc. Repeated episodes of the disease can induce complications such as gastrointestinal perforation and bleeding, affecting patients' quality of life and even endangering life safety [1]. Studies have pointed out that peptic ulcer has many causes, among which *Helicobacter pylori* (Hp) infection is the leading cause, especially in developing countries, and the infection rate is increasing year-by-year [2]. Hp, originally named *Campylobacter pyloridis*, was first identified in humans and cultured by Marshall and Warren. It is a microaerophilic, helical, gram-negative bacterium with several polar flagella for mobility. It can only survive in periplasmic pH 4.0-8.5 and can only grow in periplasmic pH 6.0-8.5 [3]. According to the survey, more than 80% of peptic ulcer patients are Hp positive. If Hp is not cleared in time, ulcer symptoms can be induced to recur, and the disease will not heal, which is not conducive to the prognosis of patients [4]. Improving the Hp clearance rate is the critical direction for the treatment of peptic ulcers. At present, quadruple therapy is the primary way to treat Hp infection-related diseases, in which the dual-use of antibiotics can enhance the antibacterial effect, which is beneficial to inhibiting the proliferation of Hp; proton pump inhibitor (PPI) can reduce gastric mucosal damage by inhibiting gastric acid secretion; bismuth is a mucosal protective agent, which is a crucial drug to promote ulcer healing [5]. Numerous studies have confirmed that quadruple therapy can improve the Hp clearance rate, reduce the risk of Hp recurrence, and elevate the clinical benefits of patients [6]. However, in recent years, studies have pointed out that some patients still experience symptoms such as acid reflux and heartburn, during drug withdrawal after quadruple therapy, which affects the therapeutic benefit to a certain extent [7]. Probiotics are defined as nonpathogenic living microorganisms that confer host health benefits when taken in moderation in food or as dietary supplements [8]. They were first proposed by Élie Metchnikoff, who theorized that Bulgarians lived longer because they consumed fermented products containing lactic acid bacteria, resulting in improved gastrointestinal health [9]. Probiotics are living microbial species with anti-inflammatory and antioxidative effects and can improve bowel microecology and general health [10]. Proper administration of probiotics is beneficial to the host. The most used probiotic bacteria are *Lactobacillus* and *Bifidobacterium* [11]. Probiotics can improve eradication of Hp and reduce side effects during therapy [12]. Probiotic supplementation aims to alter the microbiota in hopes of improving the outcome of Hp-related diseases treatment and also reducing side effects of antibiotic treatment, such as diarrhea [13]. In this study, we combined quadruple therapy with probiotics for treatment of patients with Hp-related peptic ulcers. It might provide a better treatment plan for clinical treatment of Hp-related peptic ulcers.

RETRACTED

## 2. Materials and Methods

### 2.1. General Data

A total of 180 peptic ulcer patients from May 2019 to May 2021 in BenQ Medical Center, The Affiliated BenQ Hospital of Nanjing Medical University were selected as the research subjects, and the patients and their families signed the informed consent. Inclusion criteria: (1) peptic ulcer conformed to the relevant diagnosis in the *Guidelines for Clinical Practice of Peptic Ulcer Disease* [14], and was confirmed by endoscopy; (2) the first diagnosis of peptic ulcer; (3) the Hp test result was positive; (4) all had abdominal pain, gastrointestinal bleeding symptoms; (5) quadruple therapy was performed after symptoms subside. Exclusion criteria: (1) complicated with gastrointestinal malignant tumors; (2) complicated with digestive tract obstruction; (3) complicated with Crohn's disease; (4) complicated with intestinal flora disorder; (5) continued to take antibiotics; (6) continued to take hormone drugs; (7) refractory ulcer; (8) had a history of gastrointestinal surgery. This study was approved by the medical ethics committee of the hospital. The 180 patients were divided into the study group and the control group by random number table method, with 90 cases in each group. There were no significant differences in general data including gender, age, BMI, disease site, number of lesions, and ulcer diameter between the two groups (*P* > 0.05), as shown in Table 1.

### 2.2. Treatment Methods

All patients received symptomatic treatment (such as pain relief and hemostasis) and surgical repair if necessary. After the symptoms subsided, quadruple therapy was used. The treatment methods were as follows: (1) control group: taking amoxicillin dispersible tablets (Shanxi Tongda Pharmaceutical Co., Ltd; NMPA approval number: H20000493; specification: 0.25 g) at the dose of 1.0 g/time, 2 times/d, and taking it 30 min after breakfast and dinner; taking metronidazole tablets (GrandPharma (China) Co., Ltd.; NMPA approval number: H42021947; specification: 0.2 g) at the dose of 0.4 g/time, 2 times/d, and taking it 30 min after breakfast and dinner; taking ilaprazole enteric-coated tablets (Livzon Group Livzon Pharmaceutical Factory; NMPA approval number: H20070256; specification: 5 mg) at the dose of 5 mg/time, 2 times/d, and taking it 30 min before breakfast and dinner; taking colloidal bismuth pectin capsules (Hunan Warner Pharmaceutical Co., Ltd.; NMPA approval number: H20043253; specification: 50 mg) at the dose of 200 mg/time, 2 times/d, and taking it 30 min before breakfast and dinner, for a total of 2 weeks of treatment. (2) Based on the quadruple therapy that was mentioned in the control group, the study group was supplemented with live combined *Bifidobacterium*, *Lactobacillus*, and *Enterococcus* Capsules, oral (Shanghai Shangyao Xinyi Pharmaceutical Co. Ltd.; NMPA approval number: S10950032; specification: 0.21 g/tablet) which was taken orally, 2 times/d, 2 tablets at a time.

RETRACTED

### 2.3. Observation Indicators

(1) Hp clearance rate: carbon 13 urea breath test (^13^C-UBT) was performed at the 2nd week after the treatment in the two groups to evaluate the Hp clearance rate of patients. The procedure is as follows: (1) orally taking one cup of test meal (about 12 ml); (2) collection of the exhalation at zero; (3) oral urea and start the timing. (dose: 75 mg for adults, 13C abundance >99%); (4) collecting exhalations at 10, 20, 30, 40, and 50 minutes. If the ^13^C-UBT test exceeded the benchmark value ≥ 4, it was evaluated as Hp positive. Otherwise, it was Hp negative, and the negative test result was regarded as Hp eradication. (2) Recurrence rate: ^13^C-UBT was performed at the 1st, 2nd, and 3rd months after treatment in the two groups to evaluate the Hp recurrence. During the reexamination period, Hp recurrence was used as the end event. Follow-up was stopped for patients with recurrence, and patients without recurrence continued to be followed up to the third month. (3) Gastrointestinal hormones: the 4 ml of fasting peripheral venous blood was collected before and at the end of treatment in the two groups, respectively, and centrifuged at 3500 r/min for 10 min to obtain serum (centrifugation radius was 10 cm, and the centrifuge was purchased from Nanjing Kangweida Biotechnology Co., Ltd.; model No.: Fresco 21), using radioimmunoassay (kit purchased from Wuhan Saipei Biotechnology Co., Ltd.) to detect serum gastrin (GAS), motilin (MTL), and somatostatin (SS) levels. (4) Adverse reactions: during the treatment period, the occurrence of adverse reactions, such as gastrointestinal symptoms (abdominal pain, diarrhea, nausea and vomiting, etc.), neurological symptoms (dizziness, headache, insomnia, etc.), heartburn, and acid reflux, in the two groups were observed and recorded for 2 weeks

### 2.4. Statistical Analysis

SPSS 25.0 statistical software was used to process data, % and *n*  were used to represent count data, and *χ*^2^ was used for testing. If the expected value was less than 5, continuous corrected chi-square test was used. Shapiro-Wilk normal distribution was used to test the normality of measurement data; the measurement data conforming to the normal distribution were expressed as “$\bar{x}\pm s$”, the independent sample *t*-test was used for the comparison between groups, and the paired-sample *t*-test was used for the comparison within the group. *P* < 0.05 was considered statistically significant.

## 3. Results

### 3.1. Comparison of Hp Clearance Rate and Recurrence Rate between the Two Groups

At the 2nd week after treatment, the Hp clearance rate in the study group (87.79%) was higher than that in the control group (78.89%), which was detected by ^13^C-UBT. At the 1st, 2nd, and 3rd after treatment, the recurrence rate in the study group was lower than that in the control group. At the end of follow-up, the total recurrence rate in the study group (6.67%) was lower than that in the control group (13.33%), and the difference was statistically significant (*P* < 0.05), as shown in Table 2.

RETRACTED

### 3.2. Comparison of Gastrointestinal Hormone Makers between the Two Groups

At the end of treatment, serum GAS and MTL expression decreased, and SS expression increased in the two groups compared with those before treatment. Serum gastrin and motilin expression were lower, and somatostatin expression was higher in study group than those in the control group, and the differences were statistically significant (*P* < 0.05), as shown in Table 3.

### 3.3. Comparison of Adverse Reactions between the Two Groups

There was no significant difference in the total incidence of adverse reactions including gastrointestinal symptoms, neurological symptoms, heartburn, and acid reflux between the two groups during treatment (*P* > 0.05), as shown in Table 4.

## 4. Discussion

Studies have pointed out that Hp can survive in a strongly acidic environment and is currently the only known bacterium that can survive in the stomach [15]. Hp can induce immune and inflammatory responses in the epithelial cells of the digestive tract by secreting cytotoxins, urease, lipopolysaccharide, and other proteins, which in turn lead to ulcer formation [16]. At present, Hp has been considered as a class I carcinogen, and one study has revealed that the eradication of Hp can promote the healing of peptic ulcers and prevent the malignant progression of ulcers [17]. Therefore, to promote the prognosis of peptic ulcer patients, improving the Hp clearance rate is the critical direction of clinical treatment.

Quadruple therapy, which adds bismuth to triple therapy, is currently the first-line treatment for Hp infection. Zagari et al. have demonstrated that after a 14-day treatment with quadruple therapy, the Hp eradication rate of patients is significantly higher than that of triple therapy, which effectively improves the treatment benefits of patients [18]. In this study, amoxicillin, metronidazole, ilaprazole enteric-coated tablets, and colloidal bismuth pectin capsules were used as quadruple drugs, among which amoxicillin was a *β*-lactam antibacterial drug. After oral administration, the lactam in the drug molecule can be rapidly hydrolyzed into a peptide bond, and after combining with the converting enzyme in the bacteria, it will rupture, dissolve, and lose its activity so as to play an antibacterial role [19]. Metronidazole belongs to the nitroimidazole class of antibiotics. By blocking the synthesis of cellular DNA, it interferes with bacterial growth and induces bacterial apoptosis to play an antibacterial role [20]. Studies have confirmed that amoxicillin combined with metronidazole can improve the antibacterial properties and help improve the Hp clearance rate [21]. Ilaprazole enteric-coated tablets is a second-generation PPI, which belongs to the pure levorotatory isomer of omeprazole. Since antibiotics have poor drug stability in an acidic environment, PPI can provide a favorable environment for antibiotics to function through acid suppression [22]. Bismuth has a protective effect on gastric mucosa and has been proved to have the anti-Hp effect, and its combined use with antibiotics can reduce Hp resistance to improve the antibacterial effect of antibiotics [23]. However, with the wide application of bismuth-containing quadruple therapy, the Hp resistance to related antibiotics is still on the rise, which affects the benefits of quadruple therapy to a certain extent. Khien et al. also have found that the Hp resistance to amoxicillin and metronidazole is as high as 15.0% and 69.00%, respectively, and the resistance to other antibiotics is still increasing [24]. Based on quadruple therapy, it is still necessary to continue to optimize the treatment plan and improve the Hp clearance rate to improve the prognosis of peptic ulcer patients.

RETRACTED

According to studies, peptic ulcers are still accompanied by abnormal changes in gastrointestinal hormones to varying degrees. The abnormal expression of gastrointestinal hormones can lead to mucosal damage of the digestive tract, which affects the recovery of ulcers to a certain extent [25]. GAS is a peptide substance secreted by G cells in the digestive tract mucosa. It can stimulate the secretion of hydrochloric acid and bile salts, aggravate the acidic environment of the stomach, and enhance the damage of the digestive tract mucosa. MTL is a gastrointestinal hormone secreted by Mo cells, which can aggravate ulcer disease by promoting gastric acid secretion. SS belongs to gastrointestinal hormone and neuropeptide, which can reduce gastric acid and protease secretion by inhibiting GAS secretion, which is beneficial to attenuating gastrointestinal mucosal damage and improving ulcer disease. In our study, we found that after treatment, serum GAS, and MTL expression was decreased, and SS expression was increased in the two groups compared with those before treatment. Serum GAS and MLT expression were lower, and SS expression was higher in study group than those in the control group, and the differences were statistically significant. Therefore, while treating peptic ulcers, improving the level of gastrointestinal hormones still has important clinical significance. In addition, our study indicated that there was no significant difference in the total incidence of adverse reactions including gastrointestinal symptoms, neurological symptoms, heartburn, and acid reflux between the two groups during treatment.

RETRACTED

Probiotics improves microbial balance in the intestine and plays a beneficial role for the host by preventing or alleviating intestinal infections, cancers, allergic diseases, and cardiovascular diseases [26]. Most probiotics are bacteria, with lactic acid bacteria most widely used [27]. They include *Lactobacillus* and *Bifidobacterium*, the two most common probiotics that are extensively investigated for their beneficial effects on the host. *Lactobacillus* and *Bifidobacterium* are resistant to low pH and tolerant to a wide range of temperatures as well as can promote gut maturation and integrity, protect against pathogens, and modulate the immune system [28]. In our paper, the study group was supplemented with live combined *Bifidobacterium*, *Lactobacillus*, and *Enterococcus* capsules, and this combination has been reported in treatment of irritable bowel syndrome [29]. Hp is difficult to be treated since it acquires resistance to common antibiotics. Probiotics combined with antibiotics are currently used to eradicate Hp. Probiotics are useful in treating intestinal diseases such as diarrhea. The anti-Hp activity of probiotics has also been studied [30]. The positive results of probiotics in treating Hp include improvement in eradication and tolerability. Probiotics are also good for treating Hp-related diseases. It has been documented that probiotics combined with triple therapy for treating peptic ulcer infected by Hp can greatly improve the eradication rate of Hp and increase recovery rate of patients, with less adverse reaction [31]. Several studies reveal the favorable effect of probiotics against Hp via different mechanisms including strength of mucosal barrier, competition for adhesion, and immunomodulatory mechanisms [32, 33].

Our study presents some limitations. First, we included a relatively small number of subjects in each group. In addition, there are other probiotics used to treat Hp injection besides those mentioned in this article. Therefore, more studies will be performed in the future to perfect our study.

In conclusion, based on quadruple therapy, probiotics in the treatment of Hp-related peptic ulcer patients can improve the Hp clearance rate and reduce the Hp recurrence rate, which is beneficial to improving the level of gastrointestinal hormones, with reasonable safety.

RETRACTED

## Figures and Tables

**Table 1:** General data in the two groups.

General data	Study group (*n* = 90)	Control group (*n* = 90)	Statistics	*P*
Gender [*n* (%)]				
(i) Male	58 (64.44)	50 (55.56)	*χ* ^2^ = 1.482	0.224
(ii) Female	32 (35.56)	40 (44.44)		
Age ($\bar{x}\pm s$, year)	31.88 ± 2.60	31.34 ± 2.25	*t* = 1.482	0.140
BMI ($\bar{x}\pm s$, kg/m^2^)	21.76 ± 0.69	21.71 ± 0.53	*t* = 0.501	0.617
Disease site [*n* (%)]				
(i) Gastric ulcer	68 (75.56)	58 (64.44)	*χ* ^2^ = 2.646	0.104
(ii) Duodenal ulcer	22 (24.44)	32 (35.56)		
No. of lesions [*n* (%)]				
(i) Solitary	74 (82.22)	68 (75.56)	*χ* ^2^ = 1.201	0.273
(ii) Multiple	16 (17.78)	22 (24.44)		
Ulcer diameter ($\bar{x}\pm s$, cm)	1.16 ± 0.15	1.12 ± 0.13	*t* = 1.929	0.055

**Table 2:** Hp clearance rate and recurrence rate in the two groups *n* (%).

Groups	Hp clearance rate	1st month after treatment	2nd month after treatment	3rd month after treatment	Total recurrence rate
Study group (*n* = 90)	79 (87.79)	1 (1.11)	2 (2.22)	3 (3.33)	6 (6.67)
Control group (*n* = 90)	71 (78.89)	2 (2.22)	3 (3.33)	7 (7.78)	13 (13.33)

**Table 3:** Gastrointestinal hormone makers in the two groups ($\bar{x}\pm s$).

Time	Groups	GAS (pg/ml)	MTL (ng/l)	SS (pg/ml)
Before treatment	Study group (*n* = 90)	187.24 ± 14.19	213.58 ± 15.26	26.32 ± 2.11
	Control group (*n* = 90)	184.83 ± 16.57	210.16 ± 16.64	26.78 ± 2.09
	*t*	1.735	0.566	1.245
	*P*	0.085	0.683	0.135

After treatment	Study group (*n* = 90)	92.16 ± 8.47^a^	113.25 ± 11.12^a^	49.21 ± 5.11^a^
	Control group (*n* = 90)	114.38 ± 10.02^a^	137.83 ± 12.69^a^	36.95 ± 3.91^a^
	*t*	12.311	7.267	9.364
	*P*	<0.001	<0.001	<0.001

Note: versus the same group before treatment: ^a^*P* < 0.05.

**Table 4:** Adverse reactions in the two groups *n* (%).

Groups	Gastrointestinal symptoms	Neurological symptoms	Heartburn	Acid reflux	Total incidence
Study group (*n* = 90)	3 (3.33)	2 (2.22)	1 (1.11)	1 (1.11)	7 (7.78)
Control group (*n* = 90)	1 (1.11)	1 (1.11)	2 (2.22)	1 (1.11)	5 (5.56)
*χ* ^2^					1.371^b^
*P*					0.712^b^

Note: *b* using continuous correction chi-square test.

## Data Availability

Original data included in this study can be obtained from the corresponding author under reasonable requests.

## Abbreviations

PPI: Proton pump inhibitor
Hp: Helicobacter pylori
13C-UBT: Carbon 13 urea breath test
GAS: Gastrin
MTL: Motilin
SS: Somatostatin
NMPA: National Medical Products Administration.
